The article "Heme oxygenase-1-modified bone marrow mesenchymal stem cells combined with normothermic machine perfusion to protect donation after circulatory death liver grafts" was retracted in 2022. Reasons: errors in the images; duplicated images; unreliable data.

# Heme oxygenase-1-modified bone marrow mesenchymal stem cells combined with normothermic machine perfusion to protect donation after circulatory death liver grafts

**DOI:** 10.1186/s13287-020-01736-1

**Published:** 2020-06-05

**Authors:** Huan Cao, Liu Yang, Bin Hou, Dong Sun, Ling Lin, Hong-Li Song, Zhong-Yang Shen

**Affiliations:** 1 Tianjin First Central Hospital Clinic Institute, Tianjin Medical University, Tianjin, 300070 People’s Republic of China; 2 Department of Organ Transplantation, Tianjin First Central Hospital, No. 24 Fukang Road, Nankai District, Tianjin, 300192 People’s Republic of China; 3 Tianjin Clinical Research Center for Organ Transplantation, Tianjin, People’s Republic of China; 4 NHC Key Laboratory of Critical Care Medicine, Tianjin, People’s Republic of China; 5 Tianjin Key Laboratory of Organ Transplantation, Tianjin, People’s Republic of China; 6 Key Laboratory of Transplant Medicine, Chinese Academy of Medical Sciences, Tianjin, People’s Republic of China

**Keywords:** Bone marrow mesenchymal stem cells, Donation after circulatory death, Normothermic machine perfusion, Orthotopic liver transplantation

## Abstract

**Background:**

Donation after circulatory death (DCD) liver grafts have a poor prognosis after transplantation. We investigated whether the outcome of DCD donor organs can be improved by heme oxygenase 1 (HO-1)-modified bone marrow-derived mesenchymal stem cells (BMMSCs) combined with normothermic machine perfusion (NMP), and explored its underlying mechanisms.

**Methods:**

BMMSCs were isolated, cultured, and transduced with the HO-1 gene. An NMP system was established. DCD rat livers were obtained, preserved by different methods, and the recipients were divided into 5 groups: sham operation, static cold storage (SCS), NMP, BMMSCs combined with NMP, and HO-1/BMMSCs combined with NMP (HBP) groups. Rats were sacrificed at 1, 7, and 14 days after surgery; their blood and liver tissue samples were collected; and liver enzyme and cytokine levels, liver histology, high-mobility group box 1 (HMGB1) levels in monocytes and liver tissues, and expression of Toll-like receptor 4 (TLR4) pathway-related molecules were evaluated.

**Results:**

After liver transplantation, the SCS group showed significantly increased transaminase levels, liver tissue damage, and shorter survival time. The HBP group showed lower transaminase levels, intact liver morphology, prolonged survival time, and decreased serum and liver proinflammatory cytokine levels. In the NMP and SCS groups, HMGB1 expression in the serum, monocytes, and liver tissues and TLR4 pathway-related molecule expression were significantly decreased.

**Conclusions:**

HO-1/BMMSCs combined with NMP exerted protective effects on DCD donor liver and significantly improved recipient prognosis. The effect of HO-1/BMMSCs was greater than that of BMMSCs and was mediated via HMGB1 expression and TLR4 pathway inhibition.

## Background

Liver transplantation is the most effective treatment for various end-stage liver diseases [1]. Donor graft quality can be preserved by static cold storage (SCS) using the University of Wisconsin (UW) solution [2, 3]. This solution is of great clinical significance as it increases cold ischemic tolerance of organs and has become the most widely used gold standard preservation solution for liver transplantation. However, the UW solution is associated with several shortcomings, which makes its application challenging. Researchers have developed improved storage solutions, such as histidine-tryptophan-ketoglutarate (HTK), Celsior, and Institut George Lopez solutions. The advantages of these storage solutions include improved preservation of the kidney, heart, and liver, while the disadvantages include higher occurrence of HTK-associated biliary complications. The UW solution may increase the risk of graft non-function [4]. With an increased demand for surgery, organ shortage has led to the use of extended criteria for liver donation [5–7]. Donation after circulatory death (DCD) liver grafts account for a large percentage of donor livers. According to the guidelines of the American Society of Transplant Surgeons, for DCD liver transplantation, when the actual warm ischemia time exceeds 20–30 min, the incidence of postoperative complications is significantly higher [8]. These grafts suffer serious ischemia reperfusion injury (IRI), increasing the incidence of serious complications and decreasing postoperative survival rate, which greatly affects transplantation efficiency [9, 10]. In order to improve graft quality and postoperative outcome, effective techniques to preserve DCD grafts are urgently required.

Currently, liver graft preservation methods mainly include SCS, hypothermic machine perfusion (HMP), subnormothermic machine perfusion (SNMP), and normothermic machine perfusion (NMP). SCS has failed to provide optimal DCD liver preservation, resulting in many complications. HMP may cause sinusoidal endothelial damage because it increases vascular resistance and shear stress [11]. Moreover, the liver status cannot be efficiently monitored by HMP [12, 13]. The gaseous oxygen perfusion (persufflation) technique has been shown to improve graft function after ischemic thermal injury via improving the energy status of the ischemic liver. The underlying pathways and flow patterns of persufflation require further research. However, it may pose a risk of gas embolism, and the liver status cannot be monitored during perfusion [14, 15]. Studies on SNMP are limited, and its efficacy has not been verified [16]. NMP is a novel method for in vitro liver graft preservation and offers the advantage of effective monitoring of donor liver status and protection of DCD liver [17–19]. In NMP, the liver is preserved in vitro under simulated physiological conditions, oxygen and energy are provided, normal cell physiology is maintained, and the donor liver status is monitored in real time through various physiological indicators, such as bile production and pH of the preservation solution, thus making it suitable for DCD liver preservation. NMP was previously used to perfuse the discarded DCD liver. After several hours of perfusion, recovery of cellular energy metabolism, decreased liver enzyme level, increased bile production, and restoration of liver function were observed. However, even though liver function can be restored, a liver that has undergone prolonged warm ischemia may not meet the transplantation standard [20].

In order to enhance the protective effects of NMP on organs, NMP combined with cellular therapy may be a novel strategy. Previously, some researchers used NMP to perfuse bone marrow mesenchymal stem cells (BMMSCs) into the kidney and showed that the BMMSCs could survive in the NMP system and colonize the organ [21]. Although they did not study the effect of NMP combined with BMMSCs on the kidney, they confirmed the feasibility of NMP combined with BMMSCs. In another study, researchers used NMP to perfuse genetically engineered cell sensors into the liver and showed that the engineered cells could colonize the liver, thus suggesting that this technique could be used to monitor liver status [22]. These studies confirmed the feasibility of NMP combined with cell therapy and also demonstrated the feasibility of modifying cells for organ protection in vitro. A combination of cellular therapy and NMP increases the colonization rate of cells in target organs and enhances the protective effect of NMP on such organs.

Due to their immunomodulatory functions, BMMSCs are commonly used for cellular therapy and play an important role in the study of organ damage repair and transplantation immune regulation [23]. However, BMMSC therapy has the disadvantage of insufficient migration to target organs and short survival time. Heme oxygenase 1 (HO-1), a potent cytoprotective enzyme, has been shown to exhibit antioxidant and anti-apoptotic properties, reduce cell damage, regulate immunity, and prolong the survival time of BMMSCs and enhance their activity [24–26]. In this study, HO-1-modified BMMSCs (HO-1/BMMSCs) were perfused into DCD liver grafts by NMP to increase the amount of BMMSCs in the target organ, thus enhancing their protective effect. HO-1/BMMSCs enhanced their colonization rate and survival time in target organs and enhanced the preservation of DCD liver grafts. Meanwhile, our study focused on the role of BMMSC-mediated inflammatory responses in the preservation of liver grafts.

## Methods

### Animals

All animals were obtained from China National Institutes for Food and Drug Control. Male Sprague-Dawley (SD) rats aged 3–4 weeks (40–80 g; *n* = 25) were used as a source of BMMSCs. Male SD rats aged 7–8 weeks (220–240 g) were used to establish an orthotopic liver transplantation (OLT) model. Recipients were randomly divided into 5 groups: sham operation (Sham), SCS, NMP, BMMSCs combined with NMP (BP), and HO-1/BMMSCs combined with NMP (HBP). Thirty (6 in each group) recipients were used for survival rate analysis, and the other 120 recipients were used for sample collection following OLT (naive, *n* = 6; 1 day, *n* = 6; 7 days, *n* = 6; 14 days, *n* = 6). All animals were housed in standard animal facilities for at least 3 days before use. Animals received humane care and were maintained in accordance with the guidelines established by the Committee on Laboratory Resources, National Institutes of Health. All experiments were approved by the Ethics Committee of Tianjin First Central Hospital.

### Preparation and identification of HO-1/BMMSCs

Isolation, culture, and characterization of BMMSCs were performed according to previously described methods [24, 27]. Briefly, BMMSCs were isolated from the femur and tibia of male SD rats and cultured in a cell culture incubator. Transduction was performed for third-passage BMMSCs, and adenovirus expressing HO-1 (Ad/HO-1; Jikai, Shanghai, China) was added at a multiplicity of infection of 10. The molecular biological characteristics of HO-1/BMMSCs were evaluated by in vitro osteogenic and adipogenic differentiation. Antibodies against CD29, CD34, CD45, CD90, RT1A, and RT1B (BioLegend, San Diego, CA, USA) were used for phenotype identification by flow cytometry. Immunofluorescence staining, qRT-PCR, and western blotting were used to detect the expression of HO-1.

### DCD model

The rat was anesthetized, exposing the free liver, and then, heparin (1 U/g) was injected. After 10 min of heparinization, the diaphragm was cut open and the thoracic aorta was clamped with an artery clamp; the heart was compressed to induce cardiac arrest; and the abdominal cavity was covered with 37 °C warm saline for 30 min. During this period, a temperature-sensing probe is placed in the abdominal cavity of the rat to detect and maintain the body temperature between 35 and 37 °C.

### NMP

The NMP system mainly consists of an organ chamber (capacity, 100 mL), a membrane oxygenator, a peristaltic pump, a temperature and pressure sensor, a filter, and a heat exchanger (Additional file 1). A single portal vein perfusion was performed with the perfusion temperature maintained at 36–38 °C. The total volume of perfusate was 80 mL, and the main component of the perfusate was DMEM/F12 (60 mL; Gibco, Grand Island, CA, USA) containing 20% fetal bovine serum (Biowest, Loire Valley, France). Next, 20 mL of rat blood, 100 U/mL penicillin, 100 μg/mL streptomycin, 5 U/mL heparin, 2.5 μg/mL dexamethasone, and 1 U/mL insulin were added at a perfusion flow rate of 1.5 mL/min/g, and the portal pressure was maintained at 10–14 cm H_2_O. All DCD livers were subjected to in situ flushing with 10 mL UW solution and SCS livers were stored at 4 °C for 4 h. Similarly, the NMP protocol also lasted for 4 h. The NMP livers were simply mechanically perfused. In BP group, the livers were perfused with 1.5–3 × 10^7^ BMMSCs through the portal vein. In the HBP group, the livers were perfused with HO-1/BMMSCs 1.5–3 × 10^7^. All BMMSCs were perfused into the liver through a 100-μm microthrombotic filter and stored in vitro for 4 h.

### OLT

All operations were performed by the same doctor, according to the protocol developed by Kamada and Calne [28]. The duration of the anhepatic phase was 19 ± 1 min.

### In vivo imaging

To demonstrate that BMMSCs can colonize in liver grafts, BMMSCs transfected with Ad/green fluorescent protein (GFP) (Jikai, Shanghai, China) were perfused into the liver using NMP, and liver fluorescence was measured using in an vivo imaging system on postoperative day (POD) 1.

### Biochemical examination

The levels of serum alanine aminotransferase (ALT), aspartate aminotransferase (AST), alkaline phosphatase (ALP), glutamyl transpeptidase (GGT), total bilirubin (TBil), and serum albumin were detected using an automatic biochemical analyzer (Cobas 800; Roche Diagnostics, Basel, Switzerland).

### Histology

The liver tissue was fixed in 10% neutral formalin solution, and the samples were dehydrated, embedded in paraffin, sectioned, and stained with hematoxylin and eosin (H&E). The tissue blocks were then embedded in optimal cutting temperature compound and snap-frozen in liquid nitrogen for frozen sections.

### Enzyme-linked immunosorbent assay (ELISA)

The serum was collected from the peripheral blood, and the serum levels of interleukin (IL)-1β, IL-6, tumor necrosis factor (TNF)-α, and high mobility group box 1 (HMGB1) were measured using an ELISA kit (Multisciences Biotech Co., Hangzhou, China) according to the manufacturer’s instructions.

### Immunohistochemistry and immunofluorescence

Samples were dehydrated, embedded in paraffin, sectioned, and subjected to HO-1 and cytokeratin 19 (CK19) staining (Proteintech, Wuhan, China). HO-1 staining assessments were performed using light microscopy while CK19 staining was assessed using a fluorescence microscope.

### Flow cytometry and cell sorting

Monocytes were identified in the whole blood after red blood cell lysis. The peripheral blood was incubated with anti-CD172a, anti-CD43, and anti-HMGB1 antibodies (BioLegend, San Diego, CA, USA). Flow cytometry was used to detect monocytes with high CD172a expression. Monocytes were divided into two groups of CD43^low^ and CD43^high^ monocytes based on the fluorescence intensity of CD43 [29]. The mean fluorescence intensity (MFI) of HMGB1 was measured. At the same time, CD43^low^ monocytes and CD43^high^ mononuclear cells were isolated and collected by cell sorting (FACS Aria II; BD Biosciences, Palo Alto, CA, USA).

### Western blotting

Proteins extracted from the liver tissue were analyzed by western blotting as previously described [24]. The expression of molecules related to the Toll-like receptor 4 (TLR4)/nuclear factor-κB (NF-κB) signaling pathway, such as TLR4, myeloid differentiation primary response 88 (MYD88), TNF receptor-associated factor 6 (TRAF6) (Multisciences Biotech Co., Hangzhou, China), inhibitor of NF-κB α (IκBα), phospho (p)-IκBα (p-IκBα), RelA (p65), and p-p65 (Cell Signaling Technology, Danvers, MA, USA), was detected in the liver tissue. β-actin (Multisciences Biotech Co., Hangzhou, China) was used as an internal control. Membranes were scanned with an imaging system (Bio-Rad, Hercules, CA, USA) and analyzed using Image J 7.0 software (National Institutes of Health, USA).

### qRT-PCR

Total RNA from the liver tissue was isolated using TRIzol reagent (TaKaRa Biotechnology, Japan), and cDNA was synthesized using a cDNA reverse transcription kit (TaKaRa Biotechnology, Japan) in accordance with the manufacturer’s instructions. β-actin was used as an internal control. The primer sequences are listed in Table 1.

**Table 1:** Primer sequences for qRT-PCR

Target Gene	Primer sequence	Product length (bp)
TNF-α	Forward 5′-3′:CATCCGTTCTCTACCCAGCC	146
	Reverse 5′-3′:AATTCTGAGCCCGGAGTTGG	
IL-1β	Forward 5′-3′:AGGCTGACAGACCCCAAAAG	178
	Reverse 5′-3′:CTCCACGGGCAAGACATAGG	
IL-6	Forward 5′-3′:ACAAGTCCGGAGAGGAGACT	172
	Reverse 5′-3′:TTCTGACAGTGCATCATCGC	
HO-1	Forward5′-3′:GCCCACGCATATACCCGCTAC	154
	Reverse 5′-3′:TCTGTCACCCTGTGCTTGACC	
β-actin	Forward 5′-3′:CGCGAGTACAACCTTCTTGC	200
	Reverse 5′-3′:ATACCCACCATCACACCCTG	

### Statistical analysis

SPSS 13.0 (SPSS GmbH, Munich, Germany) and GraphPad 8.0 (GraphPad Software Inc., San Diego, CA, USA) were used for statistical analysis. Data are expressed as mean ± standard deviation. Significance was tested using one-way analysis of variance. The count data were expressed as percentage (%), and significance was tested using the chi-squared test. Survival analysis using Kaplan–Meier survival curves and log-rank tests (Mantel-Cox) were performed. The Pearson correlation method was used to determine the correlation coefficient (*r*) between groups. *P* < 0.05 was considered statistically significant.

## Results

### Characterization of HO-1/BMMSCs and increased expression of HO-1 in BMMSCs after HO-1 transduction

Isolation and identification of BMMSCs was performed as previously described [30, 31]. BMMSCs transfected with Ad/HO-1 showed no morphological changes, with a typical spindle-shaped appearance (Fig. 1a), and exhibited osteogenic (Fig. 1b) and adipogenic differential potential (Fig. 1c). Flow cytometry results showed over 99% CD29, CD90, and RT1A positivity, and over 99% CD34, CD45, and RT1B negativity (Fig. 1d–f), demonstrating that Ad/HO-1 transduction did not affect the molecular biological characteristics of BMMSCs. Immunofluorescence staining results revealed the expression of HO-1 in BMMSCs (Fig. 1g) and HO-1/BMMSCs (Fig. 1h). Specifically, the red fluorescence intensity of HO-1/BMMSCs was significantly higher than that of BMMSCs. Western blot and qRT-PCR analysis (Fig. 1i) also confirmed that HO-1 expression in HO-1/BMMSCs was significantly increased.

**Fig. 1:** Characteristics of HO-1/BMMSCs in vitro and detection of HO-1 expression. **a** HO-1/BMMSCs were adherent and displayed long spindle-shaped morphology. **b** HO-1/BMMSCs showed osteogenic differentiation in vitro, as indicated by the calcareous deposits stained black with von Kossa staining. **c** Adipogenic differentiation of HO-1/BMMSCs, as indicated by oil red O-stained fat cells. **d**–**f** Surface biomarker identification. Results showed that 100.0, 99.8, and 99.4% of the cells were positive for CD29, CD90, and RT1A, respectively, and 100.0, 99.8, and 99.4% of the cells were negative for CD34, CD45, and RT1B, respectively. The molecular biological characteristics of HO-1/BMMSCs were not changed. **g** HO-1 expression in BMMSCs was identified by red fluorescence, and its intensity was weak. **h** HO-1 expression in HO-1/BMMSCs. The red fluorescence intensity was significantly higher in HO-1/BMMSCs than that in BMMSCs. **i** Western blotting and qRT-PCR results confirmed that HO-1 expression in HO-1/BMMSCs was significantly higher than that in BMMSCs

### DCD model, BMMSCs combined with NMP, and BMMSCs colonization in the liver

The normal liver had an even surface and a ruddy color (Fig. 2a), while DCD donor liver (warm ischemia time, 30 min) was dark purple-red, with an uneven surface and blunted edges (Fig. 2b). After in vitro preservation for 4 h, the SCS donor liver was slightly edematous, with blunted edges, hepatic congestion, and uneven color (Fig. 2c). The NMP, BP, and HBP livers were pale brown in color, with sharp edges and no edema (Fig. 2d–f). While NMP displayed more robust protective effects than SCS, no significant differences in liver appearance were observed between the NMP, BP, and HBP groups. Hence, a rat OLT model was successfully established (Fig. 2g–i).

**Fig. 2:** Liver appearance and colonization of BMMSCs in liver grafts. **a** The normal liver. **b** DCD donor liver (warm ischemia time, 30 min). **c** The donor liver of the SCS group was slightly edematous, with blunted edges, hepatic congestion, and uneven surface. The livers of the NMP (**d**), BP (**e**), and HBP groups (**f**) were pale brown in color, with sharp edges and no edema. **g**–**i** OLT protocol. **j** Imaging of liver grafts in vivo (**j**) and in vitro (**k**). A pseudo-color image showing the fluorescence intensity of the liver graft in vivo (**e**) and in vitro (**m**). After liver resection, no GFP fluorescence signal was detected in the rat (**n**). In the frozen liver sections, colonization of GFP/BMMSCs in the hepatic sinusoids was observed using a fluorescence microscope (**o**, × 40), indicating that BMMSCs were evenly colonized in the transplanted liver

The donor liver was perfused with GFP/BMMSCs. The BMMSCs were examined with an in vivo imaging system on POD 1. The green fluorescent signal from the liver was observed, and almost no fluorescence signal in other organs of the abdominal cavity was observed (Fig. 2j, k). Simultaneously, the pseudo-color map was used to display the fluorescence intensity. The liver fluorescence intensity was relatively uniform, indicating that the BMMSCs were uniformly colonized in the liver (Fig. 2l, m). After liver resection, no GFP fluorescence signal was detected in the rat (Fig. 2n). In the frozen liver sections, colonization of GFP/BMMSCs in the hepatic sinusoids was detected using a fluorescence microscope (Fig. 2o).

### DCD liver graft survival improved in the HBP group

The median recipient survival time was the highest in the HBP group (> 60 days) and lowest in the SCS group (2.5 days), which was significantly lower than that in the other groups (*P* < 0.05). The survival time in the BP group (37.5 days) was higher than that in the NMP group (16 days), but significantly lower than that in the HBP group (*P* < 0.05). Hence, HO-1/BMMSCs combined with NMP can significantly prolong the survival time of recipients after OLT and are more effective than BMMSCs combined with NMP (Fig. 3).

**Fig. 3:** Kaplan-Meier survival curves of OLT recipients. Median survival time of the Sham, SCS, NMP, BP, and HBP groups was > 60, 2.5, 16, 37.5, and > 60 days, respectively. Log-rank (Mantel-Cox) test results showed that the survival rate of HBP group was significantly higher than that of other liver transplantation groups (*P* = 0.0005 vs. SCS group; *P* = 0.0013 vs. NMP group; *P* = 0.044 vs. BP group)

### HO-1 expression was increased in the HBP grafts

Immunohistochemistry showed that there were greater numbers of HO-1-positive cells in the livers of the HBP group compared to those in other groups (Fig. 4A). Western blotting was used to detect HO-1 expression in the transplanted liver (Fig. 4B). Results (Fig. 4C) showed that HO-1 expression in the BP group was slightly higher than that in the SCS and NMP groups (*P* < 0.05), but significantly lower than that in the HBP group (*P* < 0.05), indicating that HO-1 transduction could improve BMMSC survival and HO-1 expression in liver grafts.

**Fig. 4:** HO-1 expression in liver grafts. **A** Immunohistochemical staining of HO-1 (× 200) showed that there were more number of HO-1-positive cells in the liver interstitial cells of the HBP group compared to that of other groups. **B** Western blot analysis of HO-1 expression. **C** Relative quantification of HO-1 protein in different groups (HO-1/β-actin) showed that HO-1 level in the HBP group was significantly higher than that in other groups (^a^*P* < 0.05 vs. SCS group; ^b^*P* < 0.05 vs. NMP group; ^c^*P* < 0.05 vs. HBP group)

### Liver function was increased in the HBP group

ALT, AST, ALP, and GGT levels were significantly higher in the SCS group than those in the other groups (*P* < 0.05). In addition, these levels were significantly lower in the BP and HBP groups than those in the NMP group at POD 7 and 14 (*P* < 0.05); however, on POD 14, the levels in the HBP group were significantly lower than those in the BP group (*P* < 0.05). These results suggested that HO-1/BMMSCs combined with NMP can improve hepatobiliary function after OLT more significantly than BMMSCs combined with NMP (Fig. 5A).

**Fig. 5:** Liver function, histopathology of liver grafts, and the Suzuki score at different time points. **A** Liver function after transplantation. On POD 1, ALT levels between the SCS (882.01 ± 139.46 U/L) and NMP groups (359.42 ± 85.13 U/L) were significantly different (*P* < 0.05), but the difference was not significant between the NMP, BP, and HBP groups (*P* > 0.05). However, on POD 1 and 7, ALT levels in the HBP (96.78 ± 35.76 U/L) and BP groups (189.46 ± 47.21 U/L) were lower than those in the SCS (395.20 ± 112.57 U/L) and NMP groups (217.46 ± 36.42 U/L), and levels in the HBP group were lower than those in the BP group. The difference was significant (*P* < 0.05), and the AST, ALP, GGT, and TBil trends were similar to ALT. **B** Pathology of liver grafts at different time points (H&E staining, × 100). On POD 1, hepatic sinusoids were enlarged and vacuolar degeneration was detected in the SCS group. A small amount of vacuolar degeneration was also observed in the NMP, BP, and HBP groups. On POD 7, partial lobular destruction was observed in the SCS group, along with liver sinus congestion and infiltration of a large number of inflammatory cells; however, these effects were improved on POD 14. The liver tissue structure was more intact in the BP group than in the SCS and NMP groups. The hepatic lobular structure of the HBP group was relatively intact, with infiltration of a small number of inflammatory cells, and its tissue structure was improved compared to that of BP group. **C** The Suzuki score at different time points (^a^*P* < 0.05 vs. SCS group; ^b^*P* < 0.05 vs. NMP group; ^c^*P* < 0.05 vs. HBP group)

### HO-1/BMMSCs combined with NMP reduced graft injury

Morphological changes were observed using H&E staining on POD 0 (naive), 1, 7, and 14. In the SCS group, on POD 7 and 14, normal lobular structure was partially destroyed and infiltration of inflammatory cells into the liver grafts was observed. The hepatic tissue structure in the BP and HBP groups was significantly improved at POD 7 and 14, and hepatic injury in the HBP group was lower than that in the BP group. These results indicated that HO-1/BMMSCs combined with NMP can improve liver graft histopathology more significantly than BMMSCs combined with NMP (Fig. 5B). The Suzuki score in the SCS group was slightly higher than that in the other groups after the preservation period. However, on POD 7 and 14, the Suzuki score in the BP and HBP groups was lower than that in the SCS and NMP groups, and the score in the HBP group was lower than that in the BP group (Fig. 5C).

Transplantation of DCD livers is associated with a high rate of biliary complications, especially ischemic cholangiopathy. Since the expression of CK19 is high in normal bile duct epithelial cells, but low in injured bile duct epithelial cells, the expression levels can be used to evaluate biliary tract injury. Immunofluorescence analyses showed greater numbers of CK19-positive cells in the livers of the HBP group compared to those in the other groups (Fig. 6A). CK19 expression in the transplanted liver was detected by western blotting (Fig. 6B). The results (Fig. 6C) showed that CK19 expression in the BP group was higher than that in the SCS and NMP groups (*P* < 0.05), but significantly lower than that in the HBP group (*P* < 0.05), indicating that HO-1/BMMSCs combined with NMP can reduce bile duct injury more significantly than BMMSCs combined with NMP.

**Fig. 6:** Expression of CK19 in biliary epithelial cells of the transplanted liver. **A** Immunofluorescence staining for CK19 (× 200, red tag) showed that the percentage of CK19-positive cells among biliary epithelial cells in the HBP group was significantly higher than that in the other groups. **B** Expression of CK19 in the transplanted liver analyzed by western blotting. **C** Relative expression of the CK19 protein (CK19/β-actin) showed that the relative expression of CK19 in the HBP group was significantly higher than that in the other groups

### HO-1/BMMSCs combined with NMP reduced the levels of IL-1β, IL-6, and TNF-α in the serum and liver tissue

The serum levels of IL-1β, IL-6, and TNF-α continued to increase at each time point in the SCS group (Fig. 7), thus being significantly higher in the SCS group than in other groups (*P* < 0.05). IL-1β and TNF-α levels in the HBP and BP groups were lower than those in the NMP group on POD 7 and 14. The proinflammatory cytokine levels in the HBP group were lower than those in the BP group on POD 14 (*P* < 0.05). The mRNA levels of IL-1β, IL-6, and TNF-α in the liver tissue were similar to the serum levels. On POD 7 and 14, the mRNA liver tissue levels of IL-1β, IL-6, and TNF-α in the HBP and BP groups were significantly lower than those in the SCS and NMP groups; however, the levels in the HBP group was lower than those in the BP group on POD 14 (*P* < 0.05). These results suggested that HO-1/BMMSCs combined with NMP can reduce proinflammatory cytokine expression more effectively than BMMSCs combined with NMP (Fig. 7).

**Fig. 7:** Levels of IL-1β, IL-6, and TNF-α in the serum and liver tissue. ELISA was used to determine the serum levels of IL-β, IL-6, and TNF-α, and qRT-PCR was used to determine the relative mRNA levels of IL-β, IL-6, and TNF-α in the liver tissue (^a^*P* < 0.05 vs. SCS group; ^b^*P* < 0.05 vs. NMP group; ^c^*P* < 0.05 vs. HBP group). On POD 1, the serum levels of IL-1β, IL-6, and TNF-α in the SCS group were significantly higher than those in other groups (*P* < 0.05), and no significant difference in levels between the NMP, BP, and HBP groups was observed. On POD 7, proinflammatory cytokine levels in the BP and HBP groups were lower than those in the SCS and NMP groups, and no significant difference in their levels between the BP and HBP groups was observed. On POD 14, their level in the HBP group decreased to near normal level and was lower than that in the BP group (*P* < 0.05). The mRNA expression pattern was similar to that of serum. The SCS group showed higher mRNA levels of IL-β, IL-6, and TNF-α than other groups on POD 1, and no difference in IL-β and TNF-α levels was observed between the NMP, BP, and HBP groups. However, on POD 7 and 14, the mRNA levels of IL-β, IL-6, and TNF-α in the BP and HBP groups were significantly lower than those in the SCS and NMP groups (*P* < 0.05), and on POD 14, their levels in the HBP group were significantly lower than those in the BP group

### HO-1/BMMSCs combined with NMP reduced serum HMGB1 levels and inhibited HMGB1 expression in monocytes and liver grafts

The serum HMGB1 levels in each group increased on POD 1, but gradually decreased to normal level in the Sham group on POD 7. However, the levels continued to increase in the SCS group and were significantly higher in this group than in other groups (*P* < 0.05). On POD 7 and 14, serum HMGB1 levels were lower in the HBP and BP groups than those in the NMP group, and on POD 14, the levels were lower in the HBP group than those in the BP group (*P* < 0.05; Fig. 8A). Flow cytometry results showed that HMGB1 expression in CD43^low^ and CD43^high^ monocytes was similar. The MFI of HMGB1 on monocytes in all groups increased on POD 1, but the increase was significantly higher in the SCS group compared to that in the other groups (*P* < 0.05). On POD 7 and 14, the MFI of HMGB1 on monocytes in the SCS group continued to increase and was higher than that in the NMP group (*P* < 0.05); however, on POD 14, the MFI of HMGB1 in the HBP group increased slightly but was lower than that in the BP group (*P* < 0.05; Fig. 8B–C3). Correlation analysis showed a strong positive correlation between serum HMGB1 level and monocyte HMGB1 expression (*r* = 0.7931; *P* < 0.0001) (Fig. 8D).

**Fig. 8:** Serum HMGB1, MFI of HMGB1 on monocytes, and HMGB1 expression in liver grafts. **A** Serum HMGB1 level. The serum HMGB1 level in the HBP group was lower than that in the SCS, NMP, and BP groups (P < 0.05). **B** MFI of HMGB1 expression on CD43^low^ monocytes (blue) and CD43^high^ monocytes (yellow). **C1** MFI of HMGB1 on CD43^low^ monocytes. **C2** MFI of HMGB1 on CD43^high^ monocytes. **C3** The MFI of HMGB1 on all monocytes in the HBP group decreased slowly after an increase on day 1, stabilized to near-normal levels on day 14, and was lower than that in the BP group (*P* < 0.05). The MFI of HMGB1 on all monocytes in the SCS group was significantly higher than those in the other groups at each time point (*P* < 0.05). **D** Correlation analysis. A strong positive correlation was observed between serum HMGB1 levels and the MFI of HMGB1 on all monocytes after OLT (*r* = 0.7931, *P* < 0.0001). **E** The protein expression of HMGB1 in monocytes and liver tissues. (^a^*P* < 0.05 vs. SCS group; ^b^*P* < 0.05 vs. NMP group; ^c^*P* < 0.05 vs. HBP group)

Western blotting was used to detect HMGB1 expression in the two monocyte groups (Fig. 8E). HMGB1 expression in the BP and HBP groups was significantly lower than that in the SCS and NMP groups on POD 7 and 14, and its expression was lower in the HBP group than that in the BP group on POD 14 (*P* < 0.05).

HMGB expression in the liver tissues of BP and HBP groups was significantly lower than that in the liver tissues of SCS and NMP groups on POD 7 (*P* < 0.05; Fig. 8E), while on POD 14, it was lower in the HBP group than that in the BP group (*P* < 0.05). These results indicated that HO-1/BMMSCs combined with NMP can reduce serum HMGB1 level and inhibit HMGB1 expression in monocytes and liver grafts more effectively than BMMSCs combined with NMP.

### HO-1/BMMSCs combined with NMP reduced the expression of TLR4/NF-κB pathway-related molecules

Expression of key molecules in the TLR4/NF-κB pathway was evaluated (Fig. 9A). On POD 7, the levels of TLR4 pathway-related molecules (TLR4, MYD88, TRAF6, p-IκBα, and p-p65) in the HBP and BP groups were significantly lower than those in the SCS and NMP groups, while their levels in the HBP group were lower than those in the BP group on POD 14 (*P* < 0.05; Fig. 9B). Hence, HO-1/BMMSCs combined with the NMP can regulate TLR4 pathway activation in the liver tissue for a long time after OLT, suggesting that they have a stronger and more prolonged inhibitory effect on the TLR4 pathway than BMMSCs combined with the NMP.

**Fig. 9:** Western blot analysis of TLR4/NF-κB signaling pathway-related molecules. **A** Expression of key molecules involved in the TLR4/NF-κB pathway as detected by western blotting. **B** Relative gray value quantitative evaluation of TLR4/NF-κB pathway-related molecules. On POD 0 (naive), the expression of molecules upstream of TLR4 was not significantly changed, but that of the downstream molecules (p-IκBα and p-p65) was altered. The expression of downstream molecules in the SCS group was higher than that in NMP, BP, and HBP groups (*P* < 0.05), but no significant difference was observed between these three groups. On POD 1, the expression of MYD88, TRAF6, p-IκBα, and p-p65 in the BP and HBP groups was lower than that in the SCS and NMP groups (P < 0.05), but no difference in expression was observed between the BP and HBP groups. On POD 7 and 14, the expression of TLR4 pathway-related molecules (MYD88, TRAF6, p-IκBα, and p-p65) in the HBP and BP groups was significantly lower than that in the SCS and NMP groups, and its expression in HBP group was lower than that in BP group (*P* < 0.05). (^a^*P* < 0.05 vs. SCS group; ^b^*P* < 0.05 vs. NMP group; ^c^*P* < 0.05 vs. HBP group)

## Discussion

BMMSCs exert their paracrine effects on organ damage repair and microenvironmental and immune regulation [32] and have been shown to promote organ and tissue repair [33–35]. However, BMMSC therapy is limited by low colonization rate and short survival time post transplantation. In addition, injection of BMMSCs into the peripheral blood may cause pulmonary embolism [36]. The HO-1 gene has been shown to enhance BMMSC activity, prolong stem cell function, and enhance liver graft preservation [24]. Here, we established a stable and reliable NMP system to enhance BMMSC colonization in the liver, thus avoiding the possible occurrence of pulmonary embolism caused by systemic application of BMMSCs. Meanwhile, our results demonstrated that BMMSC survival in the liver grafts was increased by HO-1. Moreover, BMMSCs exert protective effects on DCD liver grafts by regulating immune and inflammatory responses. However, the defect of DCD liver was a higher rate of biliary complications, including ischemic cholangiopathy. The ischemia time of DCD liver was a negative factor. Our study showed that the hepatic tissue and bile duct of BP and HBP groups was better than that of SCS and NMP groups, with the findings for the HBP group being significantly better than those for the BP group; simultaneously, BMMSCs combined with NMP to protect DCD donor liver can effectively improve the prognosis and survival of transplant recipients, and the protective effect of HO-1/BMMSCs is higher than that of BMMSCs. With the assist of NMP and HO-1/BMMSCs, the complications of using DCD liver were obviously decreased.

Next, we found that inflammation in the HBP liver was significantly reduced, as indicated by the low levels of the pro-inflammatory cytokines, IL-1β, IL-6, and TNF-α, in the serum as well as the liver tissues, indicating that HO-1/BMMSCs combined with NMP can inhibit the mRNA expression of inflammatory factors in liver grafts. HMGB1 is a proinflammatory mediator in the extracellular environment [37, 38]. We detected a rapid increase in serum HMGB1 levels. HMGB1 levels in the BP and HBP groups increased transiently after surgery and decreased at POD 7 and were significantly lower than those in the SCS and NMP groups. Since peripheral blood mononuclear cells can actively secrete HMGB1 in the serum [37, 38], we found that HMGB1 expression in monocytes after transplantation was significantly lower in the HBP groups than that in the SCS group. Moreover, HMGB1 expression in monocytes showed a strong positive correlation with serum HMGB1 content. Simultaneously, HMGB1 expression in the liver graft was significantly lower in the BP and HBP groups than that in the SCS group and was significantly lower in the HBP group than that in the BP group. These results indicated that HO-1/BMMSCs combined with NMP can significantly reduce HMGB1 liver tissue levels more effectively than BMMSCs combined with NMP. Further studies on the mechanism by which HMGB1 affects liver inflammatory responses are required.

Since HMGB1 is an important ligand of TLR4 [39], it binds to and activates TLR4 and its downstream signaling pathways. The TLR4 pathway plays a key role in regulating hepatic inflammatory response [40, 41]. Studies have shown that the absence of TLR4 in the donor organ reduces IRI in liver transplantation [42]. Clinical studies have shown that TLR4 is significantly activated in patients with IRI [43]. Therefore, studying the expression of TLR4 is very important for clarifying the protective mechanism of BMMSCs in the DCD donor liver. After HMGB1 stimulation, TLR4, an important transmembrane protein, recruits MYD88 and accepts TRAF6, releases NF-κB from the IκB/NF-κB compound migrating into the nucleus, and induces the expression of inflammatory factors, such as IL-1β, IL-6, and TNF-α [44]. In our study, we found that the protein expression of TLR4, MYD88, and TRAF6 in the liver grafts and the phosphorylation levels of the downstream molecules p-IκBα and p-NF-κB were significantly increased in the SCS group, but not in the HBP group. This suggests that the combination of HO-1/BMMSCs and NMP can prolong the downregulation of TLR4/NF-κB pathway-related molecules. Hence, in this study, we report a possible mechanism by which HO-1/BMMSCs combined with NMP protects the transplanted liver from inflammatory injury, and further demonstrate that HMGB1 plays an important role in liver graft preservation and is a key molecule of the TLR4 pathway.

In conclusion, our study showed that HO-1/BMMSCs combined with NMP can regulate HMGB1 expression in monocytes and liver grafts, thereby affecting the TLR4 pathway, inhibiting inflammatory responses, and reducing liver damage. HO-1/BMMSCs exert prolonged protective effects on liver grafts after OLT, indicating the significance of expanding the use of marginal donor livers. However, we did not perform any pathway blocking experiments and only demonstrated the role of monocytes. Our team previously studied the role of stem cells in the functioning of the corresponding immune cells of the innate and adaptive immunity in transplant recipients [30, 45]. In future, we aim to study the role of other immune cells by blocking major signaling pathways.

Although, through our research, some progress has been made in proving the efficacy of NMP combined with BMMSCs in protecting the DCD donor liver, the next step is to conduct larger animal studies for future clinical application. The NMP system established in this study has certain limitations. First, our NMP system is a single-cycle system (perfusion through the portal vein without reconstruction of the liver artery), and it is necessary to establish a double-circulation method to perfuse the human donor liver [46]. Moreover, the perfusion path of BMMSCs also requires further investigation. Secondly, the perfusate used in this study is suitable for small animal models. For clinical application, the composition needs to be improved, and a gold standard for perfusate composition for DCD liver preservation needs to be formulated. Thirdly, due to the uncertainty of the time of donor liver acquisition, BMMSCs may need to be cryopreserved. However, they display lower activity after recovery and transportation is a challenge. Hence, it is necessary to study the mechanism by which BMMSCs protect organs, and test the use of intermediate products, such as extracellular vesicles or cytokines combined with NMP for the preservation of donor liver in vitro. After several improvements in NMP combined with cellular therapy, it is believed to have broad prospects in clinical application, and may play a crucial role in expanding the donor pool and alleviating organ shortage.

Currently, NMP technology has gained much attention. In combination with other treatments, it can be used for resuscitation of marginal donor liver in vitro. In this study, HO-1/BMMSCs combined with NMP was used to preserve the DCD donor liver, thus overcoming the short survival time of BMMSCs, and improving donor liver quality and postoperative survival rate. We hope that NMP can be applied in clinical conditions, providing a new direction for the preservation and resuscitation of DCD donor livers in the future.

## Conclusions

In summary, we established a stable and reliable NMP system to enhance BMMSC colonization in the liver, thus avoiding the possible occurrence of pulmonary embolism or other complications caused by systemic application of BMMSCs. Additionally, our results demonstrated that HO-1/BMMSCs combined with NMP exerted protective effects on DCD donor livers and significantly improved recipient prognosis. The effect of HO-1/BMMSCs was greater than that of BMMSCs and was mediated via TLR4 pathway inhibition. These data are of great significance for resuscitation of marginal donor liver in vitro and expansion of donor liver pool.

## Supplementary information

**Additional file 1.** A schematic diagram of the NMP system. A stable NMP system was established. It mainly consisted of an organ chamber (aperture: 100 μm, BMMSCs and red blood cells can pass freely), a membrane oxygenator, a peristaltic pump, a temperature and pressure sensor, a filter, and a heat exchanger. Individual portal perfusion, bile duct intubation, and continuous bile production during perfusion were observed.

## Data Availability

Not applicable.

## Abbreviations

ALP: Alkaline phosphatase
ALT: Alanine aminotransferase
AST: Aspartate aminotransferase
BMMSCs: Bone marrow mesenchymal stem cells
CK19: Cytokeratin19
DCD: Donation after circulatory death
ELISA: Enzyme-linked immunosorbent assay
GFP: Green fluorescent protein
GGT: Glutamyl transpeptidase
H&E: Hematoxylin and eosin
HMGB1: High-mobility group box 1
HMP: Hypothermic machine perfusion
HO-1: Heme oxygenase-1
HTK: Histidine-tryptophan-ketoglutarate
IL: Interleukin
IRI: Ischemia reperfusion injury
IκBα: Inhibitor of NF-κB α
MFI: Mean fluorescence intensity
MYD88: Myeloid differentiation primary response 88
NMP: Normothermic machine perfusion
OLT: Orthotopic liver transplantation
POD: Postoperative day
SCS: Static cold preservation
SNMP: Subnormothermic machine perfusion
TBil: Total bilirubin
TLR4: Toll-like receptor 4
TNF: Tumor necrosis factor
TRAF6: Tumor necrosis factor receptor associated factor 6
UW: University of Wisconsin
